# Low concentration of rutin treatment might alleviate the cardiotoxicity effect of pirarubicin on cardiomyocytes via activation of PI3K/AKT/mTOR signaling pathway

**DOI:** 10.1042/BSR20190546

**Published:** 2019-06-25

**Authors:** Junjie Fei, Yi Sun, Yuyin Duan, Jianming Xia, Songhua Yu, Peigang Ouyang, Teng Wang, Guimin Zhang

**Affiliations:** Department of Cardiovascular Surgery, Affiliated Cardiovascular Hospital of Kunming Medical University, Yunnan 650032, China

**Keywords:** cardiomyocytes, cardiotoxicity effect, pirarubicin, rutin

## Abstract

Cancer is the leading cause of deaths around the world, especially in low- and middle- income countries. Pirarubicin (THP) is an effective drug for treatment of cancer, however, there still exists cardiotoxic effects of THP. Rutin is a kind of antioxidative compound extracted from plants, and might be a protective compound for cardiomyocytes. Phosphatidylinositol 3-hydroxy kinase (PI3K)/protein kinase B (AKT)/mammalian target of rapamycin (mTOR) signaling pathway is critical for cellular survival, proliferation and metabolism, and thus we speculated rutin might perform a protective role in cardiomyocytes via PI3K/AKT/mTOR signaling pathway. And in this experiment, we first established a cardiotoxicity model of THP in mice model and cell models, and then found that rutin treatment could increase the proliferation of cells at low concentration. Then we explored the possible mechanism of the protective effect of rutin using Western blotting, quantitative polymerase chain reaction (qPCR) and ELISA methods, and found that the activation of PI3K/AKT/mTOR/nuclear factor-κB (NF-κB) signaling pathway was increased, and expression of downstream molecules involved in antioxidative stress were also increased. We further noticed that concentration of angiogenesis promoting factors were also increased in medium of cultured cells. Thus, we speculated that rutin could increase the activation of PI3K/AKT/mTOR signaling pathway, further decrease the oxidative stress level via increasing the expression of antioxidative stress enzymes with the increasing concentration of angiogenesis promoting factors, resulting in the protective role in cardiomyocytes and cardiac function.

## Introduction

The mortality of cancer has been growing widely, and new cancer cases have been reported to increase to 19.3 million in 2025. Among them, more than a half of these cases will occur in low- and middle-income countries [1]. Treatments for cancer nowadays include surgery, radiotherapy, cytotoxic chemotherapy, hormonal therapy, immunotherapy, and targeted therapies [2]. However, the effect of these treatments is still limited. Pirarubicin (THP) is a new anthracycline anticancer drug which could generate cell cycle. THP alone or combined with other anticancer drugs based on THP has been proven as an effective treatment for HCC and other cancers, and presented lower cardio toxicity, faster cellular uptake, and plasma clearance [3]. However, THP and other low-molecular weight anticancer drugs could lead to severe side effects. Rutin is a flavonol glycoside composed of quercetin and disaccharide rutinose, which is produced by consumption including buckwheat groats, vegetables, and fruits. Previous studies found that rutin performed multiple pharmacological functions including antioxidant, anticarcinogenic and cardio-protective [4]. Rutin could also prevent oxidative stress via inhibiting the enzymes participating in ROS generation, such as NADPH oxidase and xanthine oxidase [5]. A previous study [10] found that rutin could prevent the cardiomyocytes from the cellular toxicity of THP via transforming growth factor-β (TGF-β1)-p38 MAPK signaling pathway, however, the detailed mechanism is not fully understood. The protein kinase B (AKT) serine/threonine kinase regulates cell survival, proliferation, growth, apoptosis and cellular metabolism. Activation of AKT by phosphorylation on Thr^308^ or Ser^473^, further phosphorylates multiple downstream proteins, including GSK3β, Bcl-2-associated death promoter, and mouse double minute 2 homolog [6]. Phosphorylated AKT could regulate apoptosis, proliferation, and cell motility via activation of mammalian target of rapamycin (mTOR) [7]. In the present study, we established cardiotoxicity model of THP in both mice model and cell model, and found that cellular proliferation and cardiac function was inhibited with THP treatment, while low concentration of rutin treatment could reverse these changes. We further found that the activity of phosphatidylinositol 3-hydroxy kinase (PI3K)/AKT/mTOR signaling pathway was increased, and the expression of antioxidative enzymes were also increased. Besides, we also found that the concentration of angiogenesis factors in cultured medium were increased. These results indicated that low concentration of rutin treatment could increase the proliferation of cardiomyocytes via PI3K/AKT/mTOR signaling pathway and the expression of downstream molecules.

## Materials and methods

### Materials

H-DMEM (10569010) and FBS (10100147) were purchased from Thermo (NY, U.S.A.). THP (72496-41-4) and rutin (153-18-4) were purchased from Dahua Pharmaceutical Co., Ltd (Wuhan, China). Total RNA Extraction Kit (R1200-100T) and TaqMan One Step RT-qPCR Kit (T2210-200T) were purchased from Solarbio Science and Technology Co., Ltd (Beijing, China). Anti-HIF-1α (hypoxia inducible factor-1α) (ab1), ROS1 (ab108492), SOD1 (ab13498), Thioredoxin (TRX) (ab26320), Peroxiredoxin1 (PRX1) (ab15571), TGF-β1 (ab64715), p-AKT (ab38449), AKT (ab179463), p-mTOR (ab109268), mTOR (ab2732), p-NF-κB (nuclear factor-κB) p65 (ab222494), NF-κB (ab207297), eNOS (ab76198) antibodies were purchased from Abcam. Angiopoietin 1 (ab99972, ab213920), FGF1 (ab219636, ab223587), VEGF (ab222510) and TGF-β (ab100647, ab119558) ELISA kits were purchased from Abcam. H9c2 (GNR 5) and Ea.hy926 (GNHu39) cells were purchased from Cell Resource Center of the Chinese Academy of Sciences.

### Animals and treatment

Twelve male wild-type (WT) C57BL/6 mice (20-week-old) were obtained from Laboratory Animal Center of the Academy of Military Medical Sciences. All mice were raised in a steady environment, which was at 25°C (temperature) and 40–70% humidity with a 12-h light and dark cycle. Mice were divided into four groups, including THP treatment group (TP), blank control group (NC), THP treatment with low-dose rutin group (TL) and THP treatment with high-dose rutin group (TH). Detailed information on mice is listed in Table 1. According to previous study, THP (1.1 mg/kg) and rutin (30 mg/kg in low-dose group and 50 mg/kg in high-dose group) were injected from periotic vein daily [8,9]. And after 7 days of treatment, cardiac function of mice was measured using MPA Cardiac Function Analysis System (Gene & I ALCBIO). After that, mice were killed using cervical dislocation and collected the heart tissue and serum sample to perform the further experiments.

**Table 1:** Baseline characteristics of mice

	TP	NC	TL	TH	*P*-value
Age (weeks)	20.4 ± 2.2	20.6 ± 2.3	19.8 ± 1.9	20.2 ± 2.0	*P*>0.05
Weight (g)	26.7 ± 3.0	28.1 ± 3.3	25.9 ± 2.7	27.3 ± 3.1	*P*>0.05
Systolic pressure (mmHg)	118 ± 9.6	122 ± 11.3	114 ± 10.4	110 ± 8.6	*P*>0.05
Diastolic pressure (mmHg)	83 ± 7.0	87 ± 8.0	82 ± 7.5	80 ± 7.1	*P*>0.05

### Cell culture, grouping, and MTT assay

H9c2 and Ea.hy 9926 cells were cultured in H–DMEM containing 10% FBS with a humid, 37°C supplied with 5% CO_2_ atmosphere. Cells were seeded into a 100-mm plate at a concentration of 1 × 10^6^, then cultured for 24 h before performing the following experiments. Cells were seeded into each well of a 96-well plate, and cultured for 24 h. According to previous study, H9c2 and Ea.hy926 cells were first treated with 5 μM THP for 24 h [10], and then they were treated with 10, 30, 50, 70 μM rutin for 1 h. After treatment, cells were incubated with MTT for 4 h at a concentration of 0.5 mg/ml. Then cells were incubated with 150 μl DMSO followed with low-speed shaking for 10 min. Optical density (OD) value at 490 nm was measured using a microplate reader. Viability rate was calculate using following equation: Viability rate = (OD_Sample_ − OD_Blank_)/(OD_Control_ − OD_Blank_) × 100%. Each experiment was repeated for three times independently.

### Evalution of cardiac function of mice using echocardiography

Cardiac function of mice was measured using echocardiography (Vevo 2100). Mice in each group were first sedated with 1.5% isoflurane anesthesia through nose cone, until successful anesthesia. Then, chest hair was removed, and cardiac function was detected using a 15-MHz probe which was placed in the parasternal, short-axis orientation. Parameters acquired under M mode were analyzed for left ventricular (LV) short axis shortening (LVFS%), LV ejection fraction (LVEF%) and LV in LV short axis (SAX) and LV long axis (PSLAX) views.

### RNA extraction and real-time quantitative polymerase chain reaction

RNA extraction was performed according to the protocol. Briefly, cells were lysed with lysis buffer, and incubated at room temperature for 5 min. Then, samples were mixed with chloroform with acute shaking for 15 s and then incubated at room temperature for 5 min. After incubation, samples were centrifuged at 12000 rpm for 10 min at 4°C, samples in water phase were collected after centrifugation. Samples were absorbed into adsorption column after centrifugation, and eluted with elution buffer after washing with washing buffer. Concentration of RNA was determined using Nano-drop 2000. Equal amount of RNA was used to perform quantitative polymerase chain reaction (qPCR) assay. Briefly, reaction mixture was made according to the protocol, and primers used are listed as follows: for H9c2 cells: caspase-3: Forward: 5′-GAGCTTGGAACGCGAAGAAA-3′, Reverse: 5′-AGTCCATCGACTTGCTTCCA-3′; caspase-9: Forward: 5′-CCACCTTCCCAGGTTTTGTCT-3′, Reverse: 5′-TCTCAGAAACAGCATTGGCGA-3′; Bax: Forward: 5′-GTTTACCTACTCGTCTCTGGTAC-3′, Reverse: 5′-CCTTATCCCAATACGTGTCGACATCAT-3′; Bcl-2: Forward: 5′-TGACGAGACCTCTATGCCGACTC-3′, Reverse: 5′-ACTTCTCATCGTACTCCCCTG-3′. And primers for Ea.hy 926 cells: caspase-3: Forward: 5′-AAATACCAGTGGAGGCCCGACTT-3′, Reverse: 5′-AAGCTTGTCGGCATACTGTTTCA-3′; caspase-9: Forward: 5′-TCTGGAGGATTTGGTGATGTC-3′, Reverse: 5′-CATTTTCTTGGCATCAGGTC-3′; Bax: Forward: 5′-CGACTACCACTTCGCCGAC-3′, Reverse: 5′-CCGTTCTGTCACTAACTTATGTTTT-3′; Bcl-2: Forward: 5′-GCTTCCCAGTCAGTCCAACA-3′; Reverse: 5′-TAACTGGTGCCTGTAGTATC-3′.

The reaction was performed under following conditions: reverse transcription: 50°C for 20 min; denaturation at 95°C for 3 min; denaturation at 95°C for 15 s, annealing at 60°C for 30 s, extension at 72°C for 45 s, these three steps were repeated for 45 cycles. The threshold cycle (*C*_T_) was calculated with normalized fluorescence signal after generation of real-time amplification. Relative analysis on expression of each gene was performed using 2^−ΔΔCq^ method according to previous study [11]. GAPDH mRNA was used as an internal reference.

### Protein extraction

Cells and mice were grouped and treated as previously described. Cells and cardiomyocytes tissues were lysed with lysis buffer (8 M Urea, 50 mM IAA, 10 mM DTT and proteinase inhibitor cocktail) on ice with ultra-sonication for 10 min. Lysis buffer was centrifuged at 12000 rpm (4°C) for 10 min, then supernatant was collected and removed into a new tube. Concentration of proteins was measured using BCA assay.

### Western blotting analysis

Sixty micrograms of protein samples were used to perform 10% SDS/PAGE electrophoresis. After electrophoresis, proteins were transferred on to a 0.22-µm nitrocellulose membrane using a semi-dry electroblotter. Membranes were incubated with primary antibodies (1:1000) overnight at 4°C, and then incubated with secondary antibody for 1 h at room temperature (1:5000). Concentration of proteins was detected using ECL immunoblotting reagent. Gray values of bands were quantitated using Scion Image software. GAPDH was used as an internal control. Each experiment was repeated for three times independently.

### Statistical analysis

Data were presented as means ± S.E.M., each experiment was repeated for three times. Differences between groups were analyzed using one-way ANOVA followed with Tukey–Kramer post hoc test. *P*-value <0.05 was set as a statistically significant difference.

## Results

### Effect of THP and rutin on cardiac function of mice

As shown in Figure 1, the LVFS% of TP, NC, TL and TH group of mice under SAX view were 24.6 ± 3.1, 63.5 ± 7.8, 51.3 ± 6.1, and 29.5 ± 4.2%, and the LVEF% under SAX view were 62.2 ± 5.6, 82.6 ± 6.1, 76.5 ± 6.0, and 57.3 ± 4.4%. The ratio of LV mass against body weight (mg/g) were 3.22 ± 0.05, 2.31 ± 0.04, 2.72 ± 0.05, and 2.76 ± 0.04. And the LVFS% of TP, NC, TL and TH group of mice under PSLAX view were 28.2 ± 3.1, 68.3 ± 5.5, 58.2 ± 4.3, and 30.2 ± 3.8%. The LVEF% under PSLAX view were 58.2 ± 5.6, 83.3 ± 7.2, 71.1 ± 6.2 and 53.2 ± 4.9. The ratio of LV mass against body weight (mg/g) were 3.35 ± 0.06, 2.85 ± 0.06, 3.12 ± 0.08, and 3.21 ± 0.07. Compared with TP group, the LVFS% and LVEF% was significantly increased in NC and TL group (*P*<0.05), while not significantly changed in TH group, and compared with NC group, the LVFS% and LVEF% was significantly decreased in TH group (*P*<0.05) both in SAX and PSLAX views. Compared with TP group, the LV mass/body weight was significantly decreased in other three groups (*P*<0.05), and compared with NC group, the ratio was significantly increased in TL and TH groups (*P*<0.05).

**Figure 1:** Effect of THP and rutin on cardiac function of mice model (**A**) LEVF% in TP, NC, TL and TH groups from SAX view. (**B**) LEVF% in TP, NC, TL and TH groups from PSLAX view. (**C**) LVFS% in TP, NC, TL and TH groups from SAX view. (**D**) LVFS% in TP, NC, TL and TH groups from PSLAX view. (**E**) LV mass/body weight in TP, NC, TL and TH groups from SAX view. (**F**) LV mass/body weight in TP, NC, TL and TH groups from PSLAX view. Data were presented as mean ± S.E.M. Each experiment was repeated for three times independently. *:P<0.05 vs. TP group. #: P<0.05 vs. control group. LEVF: Left ventricular ejection fraction.

### Effect of THP and rutin on proliferation of H9c2 and Ea.hy 926 cells

In order to screen the suitable concentration of THP and rutin for H9c2 and Ea.hy926 cells, we first performed the MTT assay on THP and rutin alone. As shown in Figure 2A, the viability rate of H9c2 cells under 10, 30, 50, 70 μM rutin treatment was 98.5 ± 5.1, 103.8 ± 5.7, 115.3 ± 4.9, and 92.3 ± 3.8. The viability rate of Ea.hy 926 cells under 10, 30, 50, 70 μM rutin treatment was 96.4 ± 4.3, 99.6 ± 4.6, 124.1 ± 5.2, and 89.6 ± 3.3 (Figure 2B). Compared with other groups, 50 μM rutin treatment could significantly increase the viability rate of H9c2 and Ea.hy 926 cells (*P*<0.05), and 50 μM rutin treatment could reduce the viabilty rate of H9c2 and Ea.hy 926 cells while only significantly of Ea.hy 926 cells. According to the result of MTT assay, we decided to use 50 μM as low concentration of rutin and 70 μM rutin as high concentration of rutin to perform following experiments. As shown in Figure 2C, the viability rate of H9c2 cells in TP, TL, and TH groups were 73.8 ± 4.1, 85.6 ± 4.5, and 65.2 ± 3.1, and the viability rate of Ea.hy 926 cells in these groups were 69.8 ± 4.0, 84.5 ± 4.2, and 62.1 ± 3.3 (Figure 2D). THP could significantly decrease the viability rate in H9c2 cells and Ea.hy 926 cells compared with NC group (*P*<0.05), and low concentration of rutin treatment could significantly incerase the proliferation of cells while high concentration of rutin treatment could significantly decerase the proliferation of cells (*P*<0.05).

**Figure 2:** Effect of THP and rutin on proliferation of H9c2 and Ea.hy 926 cells (**A**) Effect of different concentrations of rutin on cell viability of H9c2 cells. (**B**) Effect of different concentrations of rutin on cell viability of Ea.hy 926 cells. (**C**) Cell viability rate of H9c2 in different groups. (**D**) Cell viability rate of Ea.hy 926 in different groups. Data were presented as mean ± S.E.M. Each experiment was repeated for three times independently. *: *P*<0.05 vs. TP group. #: P<0.05 vs. control group.

### Effect of THP and rutin on activity of PI3K/AKT signaling pathway of mice tissue

As shown in Figure 3, in animal models, the ratio of p-AKT/AKT in TP, NC, TL and TH groups were 0.55 ± 0.04, 0.87 ± 0.07, 0.93 ± 0.07, and 0.54 ± 0.04. Compared with TP group, the ratio of p-AKT/AKT was significantly increased in NC and TL groups (*P*<0.05), and compared with NC group, the expression was significantly decreased in TH group (*P*<0.05). The ratio of p-mTOR/mTOR in these groups were 0.32 ± 0.02, 0.88 ± 0.07, 1.22 ± 0.09, and 0.89 ± 0.07. The ratio of p-mTOR/mTOR was significantly increased in all groups compared with TP group (*P*<0.05), and was significantly increased in TL group compared with NC group (*P*<0.05). The ratio of p-NF-κB p65/NF-κB in these groups were 0.90 ± 0.07, 1.42 ± 0.11, 1.60 ± 0.12, and 0.87 ± 0.07. Compared with TP group, the ratio of p-NF-κB p65/NF-κB was significantly increased in NC and TL groups (*P*<0.05), and was significantly decreased in TH group compared with NC group (*P*<0.05). And the expression of eNOS were 0.63 ± 0.05, 1.23 ± 0.09, 1.47 ± 0.11, and 1.37 ± 0.11. Compared with TP group, the expression of eNOS were significantly increased in all group (*P*<0.05). And in Ea.hy 926 cells, the ratio of p-AKT/AKT in TP, NC, TL, and TH groups were 0.66 ± 0.04, 0.96 ± 0.06, 0.87 ± 0.06, and 0.66 ± 0.04. Compared with TP group, the ratio of p-AKT/AKT was significantly increased in NC and TL groups (*P*<0.05), and was significantly decreased in TH group compared with NC group (*P*<0.05). The ratio of p-mTOR/mTOR in these groups were 0.15 ± 0.01, 0.81 ± 0.05, 0.86 ± 0.06, and 0.82 ± 0.05. Compared with TP group, the ratio of p-mTOR/mTOR was significantly increased in other three groups (*P*<0.05). The ratio of p-NF-κB p65/NF-κB in these groups were 0.39 ± 0.03, 0.85 ± 0.06, 1.03 ± 0.07, and 0.46 ± 0.03. Compared with TP group, the ratio of p-NF-κB p65/NF-κB was significantly increased in other three groups (*P*<0.05), and compared with NC group, the ratio was significantly increased in TL group (*P*<0.05) and significantly decreased in TH group (*P*<0.05). And the expression of eNOS were 0.52 ± 0.03, 0.93 ± 0.06, 1.08 ± 0.07, and 0.76 ± 0.05. Compared with TP group, the expression of eNOS was significantly increased in other three groups (*P*<0.05), and compared with NC group, the expression of eNOS was significantly increased in TL group (*P*<0.05) and significantly decreased in TH group (*P*<0.05).

**Figure 3:** Effect of THP and rutin on activation of PI3K/AKT/mTOR signaling pathway in heart tissue of mice (**A**) Western blotting analysis on expression of p-AKT, AKT, p-mTOR, mTOR, p-NF-κB p65, NF-κB, and eNOS. (**B**) Quantitative analysis of ratio of p-AKT/AKT. (**C**) Quantitative analysis of ratio of p-mTOR/mTOR. (**D**) Quantitative analysis of ratio of p-NF-κB p65/NF-κB. (**E**) Quantitative analysis on expression of eNOS. GAPDH was used as an internal control. Data were presented as mean ± S.E.M. Each experiment was repeated for three times independently. *: P<0.05 vs. TP group. #: P<0.05 vs. control group.

### Effect of THP and rutin on expression of oxidative stress-related molecules in cells and tissues

In H9c2 cells (Figure 4), the expression level of HIF-1α in TP, NC, TL, and TH groups were 1.00 ± 0.08, 0.61 ± 0.05, 0.26 ± 0.02, and 0.97 ± 0.07. Compared with TP group, the expression level of HIF-1α was significantly decreased in NC and TL group (*P*<0.05), and compared with NC group, the expression was significantly decreased in TL group (*P*<0.05) and significantly increased in TH group (*P*<0.05). The expression of ROS1 in these groups were 0.50 ± 0.04, 0.99 ± 0.08, 0.94 ± 0.07, and 0.80 ± 0.06. Compared with TP group, the expression of ROS1 was significantly increased in all groups (*P*<0.05), and compared with NC group, the expression of ROS1 was significantly decreased in TH group (*P*<0.05). The expression of TRX in these groups were 0.40 ± 0.03, 0.84 ± 0.06, 1.14 ± 0.09, and 0.81 ± 0.06. Compared with TP group, the expression of TRX was significantly increased in all groups (*P*<0.05), and compared with NC group, the expression of TRX was significantly increased in TL group (*P*<0.05). The expression of PRX1 in these groups were 0.52 ± 0.04, 0.91 ± 0.07, 0.99 ± 0.08, and 0.87 ± 0.07. And the expressions of PRX1 were significantly increased in all groups compared with TP group (*P*<0.05). And in Ea.hy 926 cells (Figure 5), the expression level of HIF-1α in TP, NC, TL and TH groups were 1.28 ± 0.09, 0.91 ± 0.06, 0.60 ± 0.04, and 1.07 ± 0.07. Compared with TP group, the expression of HIF-1α was significantly decreased in other three groups (*P*<0.05), and compared with NC group, the expression was significantly decreased in TL group (*P*<0.05) and significantly increased in TH group (*P*<0.05). The expression of ROS1 in these groups were 0.46 ± 0.03, 0.93 ± 0.06, 1.20 ± 0.08, and 0.55 ± 0.04. Compared with TP group, the expression of ROS1 was significantly increased in other three groups (*P*<0.05), and compared with NC group, the expression level was significantly increased in TL group (*P*<0.05) and significantly decreased in TH group (*P*<0.05). The expression of TRX in these groups were 0.34 ± 0.02, 0.65 ± 0.04, 0.86 ± 0.06, and 0.28 ± 0.02. The expression level of TRX presented a similar trend as ROS1. The expression of PRX1 in these groups were 0.48 ± 0.03, 0.92 ± 0.06, 0.94 ± 0.06, and 0.56 ± 0.04. The expression of PRX1 was significantly increased in other three groups compared with TP group (*P*<0.05), and the expression of PRX1 was significantly decreased in TH group (*P*<0.05) compared with NC group.

**Figure 4:** Effect of THP and rutin on activation of PI3K/AKT/mTOR signaling pathway and expression of antioxidative stress enzymes in H9c2 cells (**A**) Western blotting analysis on expression of p-AKT, AKT, p-mTOR, mTOR, p-NF-κB p65, NF-κB, eNOS, ROS1, SOD1 PRX1, TRX, and HIF-1α. (**B**) Quantitative analysis of ratio of p-AKT/AKT. (**C**) Quantitative analysis of ratio of p-mTOR/mTOR. (**D**) Quantitative analysis of ratio of p-NF-κB p65/NF-κB. (**E**) Quantitative analysis on expression of ROS1. (**F**) Quantitative analysis on expression of SOD1. (**G**) Quantitative analysis on expression of PRX1. (**H**) Quantitative analysis on expression of TRX1. (**I**) Quantitative analysis on expression of HIF-1α. (**J**) Quantitative analysis on expression of eNOS. GAPDH was used as an internal control. Data were presented as mean ± S.E.M. Each experiment was repeated for three times independently. *: P<0.05 vs. TP group. #: P<0.05 vs. control group.

**Figure 5:** Effect of THP and rutin on activation of PI3K/AKT/mTOR signaling pathway and expression of antioxidative stress enzymes in Ea.hy 926 cells (**A**) Western blotting analysis on expression of p-AKT, AKT, p-mTOR, mTOR, p-NF-κB p65, NF-κB, eNOS, ROS1, SOD1 PRX1, TRX and HIF-1α. (**B**) Quantitative analysis of ratio of p-AKT/AKT. (**C**) Quantitative analysis of ratio of p-mTOR/mTOR. (**D**) Quantitative analysis of ratio of p-NF-κB p65/NF-κB. (**E**) Quantitative analysis on expression of ROS1. (**F**) Quantitative analysis on expression of SOD1. (**G**) Quantitative analysis on expression of PRX1. (**H**) Quantitative analysis on expression of TRX1. (**I**) Quantitative analysis on expression of HIF-1α. (**J**) Quantitative analysis on expression of eNOS. GAPDH was used as an internal control. Data were presented as mean ± S.E.M. Each experiment was repeated for three times independently. *: P<0.05 vs. TP group. #: P<0.05 vs. control group.

### Effect of THP and rutin on expression of apoptosis-related genes in H9c2 and Ea.hy 926 cells

In H9c2 cells, the expression levels of Bcl-2 in these groups were 0.34 ± 0.02, 0.82 ± 0.06, 0.76 ± 0.04, and 0.51 ± 0.03 (Figure 6A). The expression levels of Bax in these groups were 1.63 ± 0.14, 0.91 ± 0.08, 0.76 ± 0.06, and 0.95 ± 0.10 (Figure 6C). The expression levels of caspase-3 in TP, NC, TL, and TH groups were 1.82 ± 0.23, 0.83 ± 0.11, 0.91 ± 0.13 and 1.45 ± 0.19 (Figure 6E), and the expression levels of caspase-9 (Figure 6G) in these groups were 1.53 ± 0.13, 0.75 ± 0.08, 0.85 ± 0.08, and 1.08 ± 0.10. And in Ea.hy 926 cells, the expression of Bcl-2 in these groups were 0.41 ± 0.03, 1.18 ± 0.09, 0.91 ± 0.07, and 0.64 ± 0.03 (Figure 6B). And the expression of Bax in these groups were 1.48 ± 0.12, 0.59 ± 0.04, 0.74 ± 0.04, and 0.93 ± 0.06 (Figure 6D). The expression of caspase-3 were 1.72 ± 0.31, 0.67 ± 0.08, 0.78 ± 0.11, and 1.12 ± 0.10 (Figure 6F). The expression of caspase-9 in these groups were 1.42 ± 0.14, 0.54 ± 0.06, 0.67 ± 0.07, and 0.82 ± 0.07 (Figure 6H). These results show that TP treatment could significantly increase the expression of pro-apoptotic molecules with the decreased expression of anti-apoptotic molecules compared with NC and TL group (*P*<0.05), while the expression of these molecules were not significantly changed between NC and TL groups.

**Figure 6:** Detection of the expression of apoptosis-related genes in H9c2 cells and Ea.hy 926 cells (**A**) Expression level of Bcl-2 in H9c2 cells. (**B**) Expression level of Bcl-2 in Ea.hy 926 cells. (**C**) Expression level of Bax in H9c2 cells. (**D**) Expression level of Bax in Ea.hy 926 cells. (**E**) Expression level of caspase-3 in H9c2 cells. (**F**) Expression level of caspase-3 in Ea.hy 926 cells. (**G**) Expression level of caspase-9 in H9c2 cells. (**H**) Expression level of caspase-9 in Ea.hy 926 cells. GAPDH was used as an internal control. Data were presented as mean ± S.E.M. Each experiment was repeated for three times independently. *: P<0.05 vs. TP group. #: P<0.05 vs. control group.

### Effect of THP and rutin on secretion of angiogenesis-related cytokines in medium and serum samples

In H9c2 cells, the concentrations of VEGF in cultured medium in TP, NC, TL, and TH groups were 158.8 ± 13.2, 242.3 ± 16.2, 233.3 ± 14.8, and 193.5 ± 14.1 pg/ml (Figure 7A). The concentrations of TGF-β in these groups were 854.5 ± 9.6, 1208.1 ± 12.5, 1124.6 ± 10.9, and 1006.2 ± 10.3 pg/ml (Figure 7C). The concentrations of FGF1 in these groups were 413.6 ± 5.4, 654.2 ± 8.5, 613.5 ± 6.6 and 565.3 ± 7.6 pg/ml (Figure 7E). The concentrations of angiopoietin-1 (Ang1) in these groups were 1940.8 ± 18.2, 2650.3 ± 23.1, 2502.3 ± 20.8, and 2365.2 ± 21.5 pg/ml (Figure 7G). And in Ea.hy 926 cells, the concentrations of VEGF in cultured medium were 112.7 ± 7.4, 194.2 ± 13.2, 176.9 ± 10.2, and 163.5 ± 9.8 pg/ml (Figure 7B). The concentrations of TGF-β in these groups were 13.6 ± 2.2, 44.1 ± 3.2, 39.2 ± 3.8, and 28.5 ± 2.4 ng/ml (Figure 7D). The concentrations of FGF1 in these groups were 363.5 ± 3.2, 533.2 ± 5.1, 496.8 ± 4.6, and 462.1 ± 4.8 pg/ml (Figure 7F). The concentrations of Ang1 in these groups were 1544.6 ± 14.2, 1950.2 ± 18.6, 1883.5 ± 17.2, and 1730.6 ± 16.2 pg/ml (Figure 7H). The concentration of these factors in cultured medium of H9c2 cells and Ea.hy 926 cells were significantly increased in all groups compared with TP group (*P*<0.05), and compared with NC group, the concentration of these factors were significantly decreased in TL and TH groups (*P*<0.05).

**Figure 7:** Detection of the concentration of angiogenesis factors in cultured medium of H9c2 cells and Ea.hy 926 cells (**A**) Concentration of VEGF in cultured medium of H9c2 cells. (**B**) Concentration of VEGF in cultured medium of Ea.hy 926 cells. (**C**) Concentration of TGF-β in cultured medium of H9c2 cells. (**D**) Concentration of TGF-β in cultured medium of Ea.hy 926 cells. (**E**) Concentration of FGF1 in cultured medium of H9c2 cells. (**F**) Concentration of FGF1 in cultured medium of Ea.hy 926 cells. (**G**) Concentration of Ang-1 in cultured medium of H9c2 cells. (**H**) Concentration of Ang-1 in cultured medium of Ea.hy 926 cells. Data were presented as mean ± S.E.M. Each experiment was repeated for three times independently. *: P<0.05 vs. TP group. #: P<0.05 vs. control group.

## Discussion

According to previous study, more than a quarter people will be affected by cancer worldwide, and surgical removal remains a mainstay in most solid cancers [12]. Microenvironment is related to integrins and focal adhesion kinases (FAKs), membrane protrusions and degradation of extracellular matrix (ECM) is closely related to the invasion, epithelial–mesenchymal transition (EMT), and metastasis of cancer cells [13,14]. THP, a tetrahydropyranyl-derivative doxorubicin, which was first found in 1979 by Umezawa et al. [15], presented an equal or superior cytotoxicity in cultured tumor cells through inhibition of invasion, EMT, and metastasis of cancer cells with less cardiotoxicity compared with DOX [16]. Antioxidative reagents has been applied in treatment of multiple cancers, especially HCC [17]. Rutin, also called quercetin-3-rutinoside, is a natural antioxidant from plant origin, and is commonly used for the treatment of cancer, oxidative stress, and cardiovascular disorders [18]. In this study, we established a cell model of cardiotoxicity of THP in mice model, and detected the effect of THP on cardiac function. Then we established a cell model of Ea.hy 926 and H9c2 under stimulation of THP, and found that rutin could increase the proliferation of Ea.hy 926 and H9c2 cells. We also found that rutin could significantly increase the activity of PI3K/AKT/mTOR signaling pathway in heart tissues of mice and cell models. The expression of antioxidative stress- and anti-apoptosis-related molecules were also increased after rutin treatment. The secretion of angiogenesis-related cytokines in cultured medium and serum samples of mice were also increased after rutin treatment. However, the protective role of rutin was more obvious in low concentration of rutin treatment group, and the protective effect in high concentration of rutin treatment group was not obvious. Thus, we speculate low concentration of rutin treatment might perform a protective role under stimulation of THP.

AKT is known as serine/threonine kinases, which belongs to general class of AMP/GMP kinase and PKC subfamily of proteins (AGC) kinases [19]. Cell growth and proliferation is under the regulation of AKT with the interaction of mTOR complex 1 (mTORC1) and the tuberous sclerosis complex 1/2 (TSC1 and TSC2). AKT could directly phosphorylate PRAS40 at T246 site, which could facilitate phosphorylation of mTORC1 at S183 site of PRAS40. This process would lead to the phosphorylation of various substrates of mTORC1 that perform an important role in cellular proliferation, including p70 s6 kinase (p70S6K1) and eukaryotic initiation factor 4E (eIF4E) binding protein 1 (4E-BP1) [20]. We noticed that the activity of PI3K/AKT/mTOR signaling pathway was decreased in mice model treated with THP with the down-regulation of the cardiac function. We also noticed that this trend could be reversed with the treatment of low concentration of rutin, while high concentration of rutin treatment seems to be cytotoxicity, as the activity of PI3K/AKT/mTOR signaling pathway was inhibited. These trend was also found in both Ea.hy 926 cells and H9c2 cells, while cultured cells seems more tolerant to high concentration of rutin. Besides, we also detected the change in expression of downstream molecules of PI3K/AKT/mTOR signaling pathway. NF-κB plays an important role in regulation of inflammation and thus regulates pro-inflammatory and coagulatory responses in endothelial cells under stress situations [21]. Using NF-κB knockout mice model, researchers found that the permeability of endothelial was decreased, with the down-regulation in expression of thrombin–antithrombin complexes [22]. Besides, NF-κB could also increase the survival ability in endothelial cells and cardiomyocytes under LPS stimulation [23]. Previous study also indicated that the translation of NF-κB could be activated by rutin treatment via increasing the phosphorylation of p38-MAPK signaling pathway [24,25]. NO in endothelial cells were synthesized by eNOS, and the expression and activity of eNOS is largely related to the function of endothelial function. Dysfunction of eNOS caused the dysfunction of coronary and peripheral vessels, leading to the occurrence of cardiovascular events [26]. As shown in the ‘Results’ section, the expression of NF-κB and eNOS was significantly decreased after THP treatment, and recovered after low concentration rutin treatment, and decreased after high concentration of rutin treatment. These results indicated that rutin could protect the cardiac cells from THP at low concentration, while high concentration of rutin might be cytotoxic.

As is well known, oxidative stress response is the main target of rutin, thus we detected the expression of critical proteins in oxidative stress response. HIF-1α is the first identified mediator response to hypoxia in cells under oxidative stress [27]. ROS1 is a receptor tyrosine kinase (RTK), which contains an N-terminal in extracellular domain, a transmembrane region, and a C-terminal intracellular tyrosine kinase domain [28]. Expression of ROS1 has been found in epithelial cells of kidneys, reproductive organs, small intestines, heart, and lungs [29]. ROS1-deficient mice have been found infertile, which is induced by differentiation of epididymal epithelial cells causing maturation in defective sperms [30]. SOD1 is an enzyme which is ubiquitously expressed in mammalian cells and blood vessels [31]. This enzyme catalyzes the converting oxygen radicalin oxygen and H_2_O_2_ through the alternate reduction. Redox homeostasis is determined by the balance between ROS production and scavenging capacity, and dysregulation in redox homeostasis would cause cellular damage, including lipoperoxidation, nucleic acid, and structure of proteins, leading to the occurrence of neurodegenerative and cardiovascular diseases. Peroxiredoxin, thioredoxin, and thioredoxin reductase form the mammalian thioredoxin system play an important role in protecting against oxidative stress injury. Prx1 is non-seleno peroxidase, which could reduce hydrogen peroxide, organic hydroperoxides and possibly peroxynitrite, forming critical antioxidants [32]. TRX is a general protein disulfide reductase, which prevents oxidative stress in cells via the reduction of PRX [33,34]. Besides, TRX also performs an important role repairing the oxidized proteins via regulating the activity of methionine sulfoxide reductases [35]. In this study, we found that the expression of these antioxidative enzymes were decreased after THP treatment, indicating that cells in heart tissue of mice were under oxidative stress, and using cultured cells, we found that viability rate of cells were decreased with the down-regulation of the antioxidative enzymes. However, after low rutin treatment, the expressions of these enzymes were recovered to normal level, even higher than that. Thus, we speculated that rutin performs a protective role in cardiomyocytes through activating the antioxidative system.

Balance between the members of Bcl-2 family proteins is critical for the survival of cells, changing in the expression of Bcl-2 family proteins could lead to the occurrence of apoptosis. Proteins in Bcl-2 family were divided into three groups: anti-apoptotic proteins (Bcl-2, Bcl-xL), pro-apoptotic proteins (Bax, Bak) and BH-3 only proteins (Bad, Bid). In this experiment, the increase in expression of Bcl-2 and decrease in the expression of Bax could increase the survival of cardiomyocytes, presenting the protective role of low-concentration rutin treatment. Caspase cascade kinases and Bcl-2 family proteins play important role in apoptosis process. Caspase-3 is the major executive caspase in apoptosis, especially in mitochondria-dependent apoptosis pathway [36]. Caspase-3 and caspase-9 are under the regulation of Bcl-2 [37], increased expression of Bax and decreased expression of Bcl-2 could induce the release of cytochrome *c* from the mitochondria, further activates caspase-9 [38], activation of caspase-3 follows with the activation of caspase-9, finally induce the occurrence of apoptosis [39]. In this experiment, we detected the expression of apoptosis-related molecules using qPCR methods, and found that low concentration of rutin treatment could increase the expression of Bcl-2 and decrease the expression of Bax, further inhibit the activation of caspase-3 and caspase-9, resulting in the inhibition of apoptosis process in cardiomyocytes.

VEGF is a well-known endothelial-specific mitogen, which could induce the physiological and pathological angiogenesis and is controlling the regulation of vascular permeability [40], besides, VEGF is also an important factor in neovascularization of tumors [41]. FGF1 is a critical factor in regulation of adipose function and is under the regulation of PPARγ. Previous study found that white adipose tissue was impaired after knockout of FGF in mice model, and leading to the occurrence of severe diabetes, and also promotes the angiogenesis process [42]. TGF-β performs multiple function in metabolism of cells both at physiology and pathology status [43]. TGF-β promotes cellular proliferation against cell death via promoting the expression of ECM protein, increasing cell motility and invasion. Ang1 is primarily expressed in vascular endothelial cells [44], and perform an important role in vascular maintenance, homeostasis, and protection. Ang1 could neutralize the side effect induced by VEGF without affecting the promoting effect in angiogenesis [45]. Up-regulation of these factors could also phosphorylates STAT3, further inducing the nuclear translocation, DNA binding, and subsequent modulation of gene transcription in downstream molecules, including NF-κB [46]. Using ELISA experiments, we detected the concentration of these angiogenesis factors in both serum samples and cultured medium of cardiomyocytes, and found that THP could significantly decrease the concentration of these factors, and low concentration rutin treatment could recover it to the normal level. And increased expression of these factors might result the recovery of cardiac function in mice model.

In the present study, we first established a cardiotoxicity model of THP using *in vivo* and *in vitro* experiment, and found that low concentration of rutin treatment could increase the proliferation. Then we found that the activation of PI3K/AKT/mTOR/NF-κB signaling pathway was increased, and expression of antioxidative stress were also increased using Western blotting analysis. We further noticed that concentration of angiogenesis promoting factors were also increased in medium of cultured cells. Thus, we speculated that rutin could increase the activation of PI3K/AKT/mTOR signaling pathway, further decrease the oxidative stress level via increasing the expression of antioxidative stress enzymes with the increase in concentration of angiogenesis promoting factors, resulting in the protective role in cardiomyocytes and cardiac function.

## Abbreviations

AKT: protein kinase B
Ang1: Angiopoietin-1
ECM: extracellular matrix
EMT: epithelial–mesenchymal transition
HIF-1α: hypoxia inducible factor-1α
LV: left ventricular
LVEF%: LV ejection fraction
LVFS%: LV short axis shortening
mTOR: mammalian target of rapamycin
mTORC1: mTOR complex 1
NC: blank control group
NF-κB: nuclear factor-κB
OD: optical density
PI3K: phosphatidylinositol 3-hydroxy kinase
PRX1: Peroxiredoxin1
PSLAX: LV long axis
qPCR: quantitative polymerase chain reaction
SAX: LV short axis
TGF-β: transforming growth factor-β
TH: THP treatment with high-dose rutin group
THP: pirarubicin
TL: THP treatment with low-dose rutin group
TP: THP treatment group
TRX: thioredoxin
